# Does the Type of Cannula Matter? A Case Report and Review of the Evidence Regarding Steel and Plastic Cannulae With Respect to a Continuous Subcutaneous Insulin Infusion

**DOI:** 10.7759/cureus.73900

**Published:** 2024-11-18

**Authors:** Maxim J Barnett, Janna Prater, Lisa Green, Jane Mayrin

**Affiliations:** 1 Internal Medicine, Jefferson Einstein Philadelphia Hospital, Philadelphia, USA; 2 Endocrinology, Jefferson Einstein Philadelphia Hospital, Philadelphia, USA; 3 Endocrinology and Diabetes, Jefferson Einstein Philadelphia Hospital, Philadelphia, USA

**Keywords:** cannula, diabetes, hyperglycemia, infusion site, insulin pump, teflon

## Abstract

A new paradigm in the management of diabetes mellitus evolved following the introduction of continuous subcutaneous insulin infusions (CSII) into clinical practice. Outcomes include greater patient satisfaction alongside improved glycemic control. Drawbacks, however, which cannot be omitted, include patient, technology, and both patient and provider error. We present a mismatch between a patient’s total daily dosage of insulin between what was expected and what was being delivered from a pump; ultimately, this required changing the infusion site and switching the type of catheter used, with resolution and improvement in clinical and glycemic status. This case is written to provide insight into one of the many complications that may be encountered with continued same-site usage of an insulin pump; moreover, strategies for management, alongside a review of the literature, are provided.

## Introduction

The delivery of insulin has evolved from syringes and vials to prefilled pens and inhaled, intravenous, and continuous subcutaneous infusions (the latter known as an insulin pump). The first prototype of an insulin pump is credited to Dr. Arnold Kadish in 1963 and was around the size of a backpack; it was then succeeded by the "biostator" by Dr. Ernst Friedrich Pfeiffer in 1974, which allowed for continuous (albeit intravenous) glucose monitoring and the formation of a closed-loop system [1]. The first commercial CSII, however, initially called the blue brick (later termed autosyringe) was designed by Dean Kamen in 1976; this had numerous adverse effects associated with it, limiting widespread acceptance for the following decades [2]. Currently, numerous pumps are available on the market, including (but not limited to) the OmniPod, Medtronic, and Tandem. The former has the advantage of being a "tubeless" pump compared to the others.

Hybrid-closed loop (or automated insulin delivery) system consists of a pump with a battery and a reservoir requiring refilling with insulin every two to three days, the infusion set with a cannula, a continuous glucose monitoring (CGM) sensor, and a transmitter. Currently, CSII allows for two different modes, including the manual mode (consisting of predetermined basal rates) and automode (which incorporates an algorithm for automatic adjustments based on the continuous glucose monitoring).

Despite the various models and brands available, there does not appear to be a survival advantage of one pump over another [3]. Although the introduction of CSII has allowed greater patient autonomy and glycemic control, there are notable drawbacks including the risk of treatment failure. We present a case report of worsening glycemic control on an insulin pump, and the strategies involved in management, alongside a review of the literature.

## Case presentation

A 63-year-old female with latent autoimmune diabetes in adults is seen in the clinic. She was initially diagnosed with type 2 diabetes mellitus and managed on metformin; however, her glycemic control continued to deteriorate, and further investigations demonstrated positive autoantibodies. Insulin therapy with multiple daily injections was initiated. She was eventually transitioned to CSII via a Tandem insulin pump with a Dexcom G6 CGM.

In the clinic, she noted that she had recently been discharged from an outside hospital for diabetic ketoacidosis. Upon review of her CGM data, her average blood glucose was 263 mg/dL, with a time in range of 0% (more than 180 mg/dL 94% of the time). Peculiarly, despite a usual total daily dose of around 40 units, she was receiving triple this amount (128 units per day) via an insulin pump (Table 1).

**Table 1:** Comparison of glycemic values before and after site and cannula change GMI: glucose management indicator

Continued insulin infusion site	Change of site + steel infusion	Three months later
Time in range: 0%	Time in range: 38%	Time in range: 52%
Average reading: 263 mg/dL	Average reading: 202 mg/dL	Average reading: 185 mg/dL
GMI: no data	GMI: 8.2%	GMI: 7.7%
Average daily dose: 128.31 units	Average daily dose: 46.06 units	Average daily dose: 61.38 units

It was revealed that she had been using the same infusion site-her abdomen-with each new infusion set. As a result, she was advised to change the type of infusion sets and switch from a plastic to a steel infusion set due to the development of lipohypertrophy and presumed poor absorption of insulin. Upon follow-up one month later after switching to a steel infusion set and rotation of infusion sites, her pump was now administering an average of 46.06 units per day (Table 1). Glycemic control improved.

## Discussion

A true figure of the number of insulin pumps in use globally cannot be determined; however, estimates range between 750,000 and 1,000,000 [4]. Similarly, a true figure reporting the number of adverse events relating to an insulin pump is unknown. Insulin pump malfunctions may include problems with the pump itself (such as failed battery, alarm settings, and complete breakdown), delivery of the insulin (such as infusion set or cannula failure, dislodgement, and blockage), cutaneous complications (such as tunneling, lipohypertrophy, and infection), or human error related to the settings of the pump.

Insulin pump manufacturers usually recommend the cannula and catheter (tubing) be changed every three to seven days [4]. The basis for changing after three days initially stemmed from a case report in 1983 of an 11-year-old female patient who kept the same infusion set for 10 days and ultimately developed an abscess and toxic shock syndrome [5]. There is concern that after three days, the cannula will be recognized as a foreign object and commence an inflammatory cascade in the skin along with fluids attaching to cannula pores [4]. Of note, however, many patients do not adhere to changing the cannula and catheter (tubing) every three days; as presented by Wilcox et al. [6], 27% of participants were noted to wear an infusion set for more than three days. Moreover, despite the three-day recommendation, numerous authors have demonstrated that after 48 hours, there is a deterioration in glycemic control. Thethi and colleagues [7] assessed a pump infusion line for up to 100 hours, demonstrating a significant increase in all glucose domains after 48 hours (prandial, mean daily, two-hour postprandial, percentage of time above 180 mg/dL). Schmid et al. [8] followed 24 patients, noting that within two days, there were 290 catheter-related adverse events, and after four days, 495 events. van Bon et al. [9] performed a multicenter study with Teflon infusion sets for around 71 hours, observing unexpected hyperglycemia occurring in the majority of patients (61% with lispro, 62% with aspart, and 68% with glulisine).

An estimated 4.6%-15% of all infusion sets are likely to fail within three days of insertion (leading to hyperglycemia) [10]. Thethi et al. [7] noted that after wearing an infusion set for five days (with continuous glucose monitoring) in a crossover study assessing lispro and aspart, significant rises in glucose from days 2 to 5 occurred (123 mg/dL to 164 mg/dL, p < 0.05) with an increase in the total daily dose of insulin (49 +/- 12 versus 55 +/- 18, p = 0.05); in contrast, however, other studies such as that of Perrin and colleagues [10] have failed to demonstrate a significant increase in the total daily dose of insulin despite successive mean increases in glucose (126 mg/dL on day 1, 133 mg/dL on day 3, 147 mg/dL on day 5, p < 0.001).

A "silent occlusion" refers to an occlusion not initially detected by the system due to the requirement for back pressure to develop. In the study by Klonoff et al. [11], 66% of their subjects had hyperglycemia with insulin pump usage, with 36% of these recorded episodes as a result of an occlusion of the infusion. Van Bon et al. [12] assess five different insulin pumps operating at two different flow rates and purposely clipped the catheter; the time from occlusion to alarm varied from 1.5 to 24 hours, with a median of 2-4 hours. Moreover, the time for alarm occlusion was near-double for an infusion of 0.5 units/hour compared to 1.0 units/hour. Zisser [13] demonstrated an approximate 1 mg/dL per minute rise in glucose for the first half-hour following shutting off a pump, estimating that an alarm would not sound until glucose has risen by 120-240 mg/dL.

Pertaining to the case depicted above, there is concern regarding the type of cannulae used in delivering insulin. Højbjerre et al. [14] assess 10 healthy male subjects and compare tissue response and adipose tissue blood flow with Teflon and steel cannulae noting that after 48 hours, blood flow significantly increased in the Teflon with minor increase in the steel cannula (moreover, the Teflon required higher flow pressure). The authors further demonstrate mean perfusion pressure is significantly greater after 48 hours of wear time with Teflon rather than steel catheters, with greater maximal pressure required to deliver a bolus with Teflon cannulae (as well as increase in adipose tissue blood flow) [14]. One limitation to this study, however, was that it was only over 48 hours. Patel et al. [15] perform a crossover trial with both Teflon and steel infusions in 20 patients; on the first day, 15% of Teflon cannulae failed due to kinking on insertion which was recognized by hyperglycemia or a high-pressure alarm hours later. The authors state that there is no overall significant difference in body mass index in those who experienced kinking and those who did not and express that there is no difference between steel and Teflon infusions sets in function over seven days (Kaplan-Meier survival failing to demonstrate difference in failure rates). Moreover, the authors cite that the greatest predictor of function of the infusion is the subject rather than the set (87% steel and 77% Teflon were functioning after three days, 68% steel and 59% Teflon after five days, 53% and 46% after six days, and 32% and 33% after seven days). Clausen et al. [16] stated that while Teflon cannulae can increase blood flow and lead to more rapid absorption of insulin (in the first two days of wearing the catheter), there is no change in peak concentration of total insulin absorption following boluses. A study in Germany (including 432 children) is performed by Liebner et al. [17] with 56% using Teflon, and 44% using steel cannulae, presenting no difference in complications relating to materials. In another study with 40 subjects each wearing two Teflon and two steel cannulae, mild infusion site reactions are noted, without differences in skin reactions/wear time [18].

Similar to the 15% of insertion failures noted above [10], Renard et al. [19] presented a 9% failure rate on initial insertion with vertically inserted Teflon catheters, which is deemed to be due to kinking after contact with muscular fasciae. An estimated 6% of 6 mm 90-degree insertions will likely be intramuscular in adults; when compared to pediatrics, up to 38% of 6 mm needle injections will be intramuscular in ages 7-13 years and 35% in 14-17 years [20, 21]. In a meta-analysis of 25,154 infusion sets (assessing 90-degree Teflon to angled Teflon), Kanapka et al. [10] elicited higher rates of hyperglycemia in the former group at three days (4.0% versus 1.3%, p = 0.01, OR 2.0, 95% CI 1.2-3.3). Moreover, the authors compare to a steel set infusion as well, identifying a rate of hyperglycemia of 1.9% (p = 0.006, OR 1.8, 95% CI 1.2-2.8). Rabbone and colleagues [22] analyze 1,046 young patients with type 1 diabetes mellitus nearly all using Teflon infusion sets (78% 90-degrees, 22% oblique), documenting failure rates of around 7% with hyperglycemia. One benefit to 90-degree Teflon infusions, however, is the report of lower risk for local skin reactions [23].

## Conclusions

Although the advantages of insulin pumps are multifold, it is imperative for the clinician (and expert patient) to be aware of the potential for adverse events and to recognize malfunction. Presented in this report is a complication that occurs when using the same site for an insulin pump, which led to a delay in recognition and deterioration in glycemic control. A literature review is additionally presented to further enhance the understanding of this concept.
